RETRACTED

# TRB3 Is Involved in Free Fatty Acid-Induced INS-1-Derived Cell Apoptosis via the Protein Kinase C δ Pathway

**DOI:** 10.1371/journal.pone.0096089

**Published:** 2014-05-13

**Authors:** Jun Qin, Ni Fang, Jinning Lou, Wenjian Zhang, Shiqing Xu, Honglin Liu, Qing Fang, Zai Wang, Jiang Liu, Xiuli Men, Liang Peng, Li Chen

**Affiliations:** 1 Department of Endocrinology, Qilu Hospital of Shandong University, Jinan, Shandong, China; 2 Institute of Clinical Medical Sciences, China-Japan Friendship Hospital, Beijing, China; 3 Department of Neurosurgery, China-Japan Friendship Hospital, Beijing, China; 4 Department of Pathophysiology, North China Coal Medical University, Tangshan, China; Hertie Institute for Clinical Brain Research and German Center for Neurodegenerative Diseases, Germany

## Abstract

Chronic exposure to free fatty acids (FFAs) may induce β cell apoptosis in type 2 diabetes. However, the precise mechanism by which FFAs trigger β cell apoptosis is still unclear. Tribbles homolog 3 (TRB3) is a pseudokinase inhibiting Akt, a key mediator of insulin signaling, and contributes to insulin resistance in insulin target tissues. This paper outlined the role of TRB3 in FFAs-induced INS-1 β cell apoptosis. TRB3 was promptly induced in INS-1 cells after stimulation by FFAs, and this was accompanied by enhanced INS-1 cell apoptosis. The overexpression of TRB3 led to exacerbated apoptosis triggered by FFAs in INS-1-derived cell line and the subrenal capsular transplantation animal model. In contrast, cell apoptosis induced by FFAs was attenuated when TRB3 was knocked down. Moreover, we observed that activation and nuclear accumulation of protein kinase C (PKC) δ was enhanced by upregulation of TRB3. Preventing PKCδ nuclear translocation and PKCδ selective antagonist both significantly lessened the pro-apoptotic effect. These findings suggest that TRB3 was involved in lipoapoptosis of INS-1 β cell, and thus could be an attractive pharmacological target in the prevention and treatment of T2DM.

## Introduction

Beta cell dysfunction is one of major characteristics in the pathogenesis of type 2 diabetes [1]. Circulating adipose tissue-derived products such as FFAs play a direct role in pancreatic β cell dysfunction and death. A high plasma concentration of FFAs is indeed a risk factor for the development of type 2 diabetes [2]. In addition, many studies have validated that FFAs induce β cell dysfunction and apoptosis [3], [4]. However, the mechanisms underlying FFAs-induced β cell apoptosis and dysfunction are not well understood.

The Tribbles family as an inhibitor of mitosis was first described in Drosophila, and has been shown to regulate cell morphogenesis, proliferation and migration [5]–[7]. TRB3, the best studied member of the mammalian Tribbles family, coordinates crucial cellular processes, including adipocyte differentiation, lipid metabolism, regulation of collagen expression, and modulation of tumorigenesis [8]–[11]. In addition, several studies have described that TRB3 promotes apoptosis [12], [13] while others have revealed TRB3 to possess an anti-apoptotic role [14], [15]. In diabetes mellitus, besides impairing insulin action in peripheral tissues by binding and inhibiting AKT/PKB phosphorylation [16]–[18], TRB3 was reported to be involved in β cell apoptosis induced by cytokines [13]. Although a few studies have suggested a close association of TRB3 with pancreatic β cell apoptosis, the potential significance of the regulation of TRB3 function to FFAs-induced β cell apoptosis deserves further investigation.

RETRACTED

The present study was designed to identify the importance of TRB3 in lipotoxicity -induced β cell apoptosis and to investigate the relevant mechanisms underlying TRB3's activity in β cells.

## Result

### Saturated FFA, palmitate, induced apoptosis, and upregulated TRB3 expression in INS-1 cells and in mice islets

Consistent with previous studies, we found that palmitate induced apoptosis in INS-1 cells in a duration- and dose-dependent manner (Fig. 1A and B). Meanwhile, TRB3 expression was upregulated as INS-1 cells were exposed to increasing duration and concentration of palmitate (Fig. 1C and D). We injected palmitate into mice intraperitoneally once daily for 7 days, and serum free fatty acid increased markedly (Fig. 1E) without resulting in a significant increase in body weight (data not shown). In addition, caspase-3/7 activity in the isolated islets was increased in palmitate-injected mice (Fig. 1F) accompanied by a significant increased expression of TRB3 (Fig. 1G). We also injected unsaturated FFA oleate (which have been shown to lack effects on beta cell apoptosis) into mice intraperitoneally once daily for 7 days, and serum free fatty acid increased markedly (Fig. 1E). However, caspase-3/7 activity and TRB3 expression in the isolated islets were not increased in oleate-injected mice (Fig. 1F and G). In summary, we observed that TRB3 expression was upregulated upon exposure of cells to saturated FFAs, and such upregulation correlated with increased β cell apoptosis.

**Figure 1:** Saturated FFA, palmitate, induced apoptosis, and upregulated TRB3 expression in INS-1 cells and in mice islets. (A) Time-course and (B) dose-response of palmitate-induced apoptosis in INS-1 cells. To investigate the time-course of apoptosis induced by palmitate, cells were cultured in the presence of 0.2 mM palmitate for the indicated duration. To study the trend of apoptosis with changing concentrations of palmitate, cells were cultured with the indicated concentrations of palmitate for 24 h. Apoptosis was assessed by TUNEL staining, and columns represent mean ± S.E.M. of three independent experiments, each conducted in triplicate (*p<0.05, **p<0.01 ANOVA/Tukey test). Scale bar, 50 µm. (C) Time-course and (D) dose-response of palmitate on TRB3 expression in INS-1 cells were analyzed by western blot. A representative blot of 3 independent experiments is shown. C57BL/6 mice (10–12 weeks old) were intraperitoneally injected with 0.5 ml of 5 mM palmitate, oleate, or BSA (3.75%) per day for 7 days. Serum FFA levels were increased after palmitate or oleate intraperitoneal injection (E). Apoptosis in the isolated islets was assessed by caspase-3/7 activity (F). Mean ± S.E.M. of the palmitate injected groups, oleate injected groups, and control groups (BSA injected) are shown, samples were tested in triplicate (n = 5 for each group, *p<0.05, **p<0.01, unpaired two-tailed t test). (G) Expression of islet TRB3 was detected by western blot, representative blot of 3 independent experiments is shown.

RETRACTED

### Overexpression of TRB3 induced apoptosis and exacerbated lipoapoptosis

In order to investigate the exact role of TRB3 in palmitate-induced β cell apoptosis, we used a stable cell line capable of an inducible expression of TRB3, termed TRB3 cells. The cells were induced with 500 ng/ml of doxycycline (Dox) for 48 h and TRB3 expression and cell apoptosis were analyzed. As shown, Dox markedly induced TRB3 expression (Fig. 2A and 2B) and cell apoptosis (Fig. 2C and 2D). However, Dox alone did not affect endogenous TRB3 expression (data not shown) and cell apoptosis (Fig. S1) in INS-1 cell control. Then TRB3 cells were exposed to either vehicle or 0.2 mM palmitate for 24 h. The extent of apoptosis was assessed by TUNEL staining and caspase 3 activity assay. Exposure of TRB3 cells to palmitate caused moderate apoptosis. However, concomitant overexpression of TRB3 exacerbated palmitate-induced apoptosis (Fig. 2C and 2D).

**Figure 2:** Overexpression of TRB3 induced apoptosis and exacerbated lipoapoptosis. In the presence or absence of 500/ml Dox for 48 h, the response of TRB3 inducible β cell line was analyzed by western blot (A), and immunofluorescence staining (B). Values represent the mean ± S.E.M. of three independent experiments (*p<0.01 unpaired two-tailed t test), Scale bar, 100 µm. TRB3 cells were cultured with or without 500 ng/ml Dox for 48 h and then treated with or without 0.2 mM palmitate for 24 h. Cell apoptosis was induced by TRB3 overexpression and exacerbated by the addition of palmitate. Apoptosis was assessed by TUNEL staining (C) and caspase 3 activity (D). Columns represent mean ± S.E.M. of three independent experiments, each conducted in triplicate (*p<0.05, **p<0.01 ANOVA/Tukey test). Scale bar, 50 µm.

RETRACTED

### TRB3 knockdown significantly inhibited palmitate-induced apoptosis

To further demonstrate the role of TRB3 in lipoapoptosis, we knocked down TRB3 expression by siRNA in INS-1 cells. The efficiency of TRB3 silencing is summarized in Fig. 3A. As shown in Fig. 3B and 3C, TRB3 silencing largely offset the apoptotic effect of palmitate in INS-1 cells. Altogether, the data above implicated TRB3 in palmitate-induced apoptosis.

**Figure 3:** The effect of TRB3 knockdown on palmitate-induced apoptosis. Western blot was used to confirm TRB3 silencing efficiency in INA-1 cells (A). (B and C) TRB3 knockdown inhibited palmitate-induced apoptosis in INS-1 cells. After transfection with TRB3 siRNA for 2 days, INS-1 cells were treated with or without 0.2 mM palmitate for 24 hours. Cell apoptosis was assessed by TUNEL staining (B) and caspase-3 activity assay (C). Columns represent mean ± S.E.M. of three independent experiments conducted in triplicate (*p<0.05, **p<0.01, ANOVA/Tukey test). Scale bar, 50 µm.

### TRB3 mediated FFAs-induced apoptosis via PKCδ activation

Previous reports have demonstrated that TRB3 could interact with AKT and participate in cell apoptosis and insulin resistance [13], [16], [19]. We examined AKT activation in INS-1 derived cells and observed that overexpression or knockdown of TRB3 had no obvious effect on AKT activation (Fig. S2). Similar observation was reported upon genetic deletion of TRB3 in mice [20]. Therefore, we hypothesized that TRB3 mediates FFAs-induced apoptosis via a signaling pathway other than the AKT pathway.

PKCδ has been reported to play a decisive role through its nuclear translocation and kinase activity of PKCδ in β cell apoptosis induced by FFAs [21]–[23]. Besides, using our i.p injection model in Figure 1E–G, we found that palmitate not only increased TRB3 expression and apoptosis, but also promoted nuclear translocation and activation of PKCδ in isolated islets, while unsaturated FFA oleate had no such effects (Fig. S3). So we speculated that TRB3 may mediate lipoapoptosis through PKCδ pathway.

In cultured TRB3 cells, accompanied with TRB3 upregulation, PKCδ was activated and accumulated in the nuclei (Fig. 4A). Since translocation of PKCδ to the nucleus may dependent upon phospholipase C (PLC) activity in β cell lipoapoptosis [21], we initially tested the effects of the general PLC inhibitor U-73122. We found that U-73122 reduced the apoptosis restricted to TRB3 overexpression significantly (Fig. 4B), preventing nuclear accumulation of PKCδ without altering the expression of TRB3 (data not show). In addition, a similar effect was observed when rottlerin, a selective inhibitor of PKCδ [24], [25], was added (Fig. 4C). These results indicated that PKCδ is a novel and key downstream mediator of TRB3 effects in lipoapoptosis.

RETRACTED

**Figure 4:** TRB3 mediates FFAs-induced apoptosis via PKCδ activation. We investigated the nuclear translocation (nuclear PKCδ vs. nuclear H1) and activation (phosphorylated PKCδ vs. whole-cell PKCδ) of PKCδ in TRB3 cells after TRB3 overexpression (TRB3 vs. β-actin) (A). To investigate the nuclear translocation of PKCδ, the nuclear proteins were prepared using NE-PER Nuclear Protein Extraction Kit and subjected to western blots analysis using antibody against PKCδ, with Histone H1 as controls for equal loading of proteins. To investigate the phosphorylation (activation) of PKCδ, whole-cells were lysed in RIPA buffer containing protease inhibitors and phosphatase inhibitors. Whole-cell proteins were subjected to western blots analysis using antibodies against phosphor-PKCδ, with β-actin as controls for equal loading of protein. Each blot is representative of three independent experiments. TRB3 cells were pretreated with U73122 (B) or rottlerin (C) for 1 hour, and incubated with Dox (500 ng/ml, 48 h), followed by palmitate (0.2 mM, 24 h). Cell apoptosis was assessed by TUNEL staining (B and C). The bar graph shows the average apoptosis rate, values represent mean ± S.E.M. of three independent experiments, each carried out in triplicate(*p<0.05, **p<0.01, ANOVA/Tukey test), Scale bar, 50 µm.

### TRB3 mediated FFAs-induced INS-1-derived cell apoptosis *in vivo*

To validate our *in vitro* results, we transplanted TRB3 cells into the renal capsules of streptozotocin (STZ)-treated diabetic mice. Since the INS-1 cell line is derived from rat insulinoma, the cells will be xenografted in the renal capsules (Fig. 5A and B). About 2 weeks post-transplantation, the fasting blood glucose of the mice began to decline gradually (Fig. 5E). These data suggested that INS-1-derived cells as xenografts indeed secreted insulin to lower blood glucose (Fig. 5C, E and F). Then, the mice were intraperitoneally injected once daily with Dox to induce TRB3 overexpression (Fig. 5D) and with palmitate to increase the plasma FFAs. After 8 days, the groups treated with Dox or palmitate exhibited increased blood glucose levels, which were further enhanced in the group treated with both Dox and palmitate. We supposed that differences in blood glucose between the groups were due to the activity of TRB3 on cell apoptosis varying in the presence or absence of palmitate. To confirm our speculation, we assessed the apoptosis in TRB3 cell xenografts by TUNEL staining (Fig. 5G) for each treatment group. As expected, TRB3 overexpression exacerbated FFAs-induced apoptosis.

RETRACTED

**Figure 5:** TRB3 mediated FFAs-induced INS-1-derived cell apoptosis *in vivo*. (A) Representative images of the kidney of nu/nu mice in each experimental group. (B) Example of H&E stained images, and (C) immunohistochemical staining for insulin in xenografts. (D) Immunohistochemical staining for TRB3 in xenografts of each group. (E) Average fasting blood glucose levels of the 4 experimental groups (controls, mice treated with Dox, mice treated with palmitate, mice treated with a combination of Dox and palmitate). (F) Average fasting plasma insulin levels at the end of the experiments and (G) apoptosis in xenografts, as assessed by TUNEL staining. (H) Blocking PKCδ activation by rottlerin inhibited TRB3-mediated β cell apoptosis under high plasma FFAs conditions *in vivo*. From day 18 after transplantation of TRB3 cells, mice were intraperitoneally injected with rottlerin to inhibit PKCδ activity and Dox to induce TRB3 expression, and then treated with or without palmitate. Apoptosis in xenografts assessed by TUNEL staining. Data shown are expressed as mean ± S.E.M (*n* = 6, *p<0.05, **p<0.01). Scale bar, 50 µm.

Using the animal model described above, we further assessed whether blocking PKCδ activation by rottlerin could inhibit TRB3-mediated β cell apoptosis under high plasma FFAs conditions *in vivo*. As shown in Fig. 5H, injections of rottlerin (0.3 mg/kg) inhibited PKCδ phosphorylation, which significantly prevented TRB3-mediated β cell apoptosis under high plasma FFA conditions. These results indicate that TRB3 could activate PKCδ and mediate FFAs-induced INS-1-derived cell apoptosis *in vivo*.

## Discussion

Accumulating evidence indicate that FFA are chronically elevated in obesity-linked T2DM. Numerous *in vivo* and *in vitro* studies have demonstrated the destructive effects of chronic exposure of FFA on β cell survival T2DM is characterized by peripheral insulin resistance and pancreatic β cell dysfunction resulting in defective glucose-induced insulin secretion and β cell dysfunction and loss through apoptosis [3], [4], [26] which is thought to largely contribute to development and progression of T2DM. Although the overall picture is known, mechanisms of lipoapoptosis in β cells are still very fragmentary and the details remain to be further examined. This study was designed to identify the mechanisms of lipotoxicity in diabetes and to test the hypothesis that TRB3 may play a critical role in apoptosis of β cells induced by FFAs.

RETRACTED

In the present study, we demonstrated that TRB3 is indeed expressed in pancreatic β cells, hence providing an avenue for deciphering its role in the pathogenesis of diabetes. The expression of TRB3 became significantly elevated in mice islets and in INS-1 β cells under FFAs stimulation, and it correlated with increased cell apoptosis. Moreover, we also found that FFAs-induced apoptosis was enhanced by TRB3 overexpression, while inhibited by TRB3 silencing. These results confirmed our speculation that TRB3 plays an important role in FFAs-induced apoptosis. Furthermore, we confirmed the effects of TRB3 on FFAs-induced β cell apoptosis *in vivo* for the first time, using a sub-renal capsular transplantation animal model. Importantly, this animal model offers a new option for studying gene function in INS-1 cells *in vivo*.

The mechanisms underlying TRB3 involvement in FFAs-induced apoptosis were further examined. The discovery of TRB3 action on β cell apoptosis and insulin resistance highlighted the specific significance of AKT pathway [18], [27]. However, this has recently been challenged. Okamoto et al. found that genetic deletion of TRB3 in mice failed to alter AKT activation [20] and Iynedjian et al. reported that overexpression of TRB3 had no effect on inhibiting AKT-mediated insulin signaling in hepatocytes [28]. We examined AKT activation in INS-1 derived cells and observed that overexpression or knockdown of TRB3 had no obvious effect on AKT activation, suggesting a minor role of AKT in our cell system. Therefore, we hypothesized that TRB3 mediates FFAs-induced apoptosis via a novel signaling pathway other than the AKT pathway.

Several isoforms of protein kinase C family have been shown to be involved in the fatty acid-dependent signaling. PKCδ, one of the novel isoforms of PKC, was shown to exert anti-apoptotic and -proliferative effects in various cell types. As one of the more abundantly expressed isoforms in β cells, PKCδ, favors β proliferation through phosphorylation p21^Cip/WAF^ which result in nuclear extrusion of the cell cycle inhibitor under stress-free conditions [23]. Under stress conditions, PKCδ has been identified as a promoter in β apoptosis [29], [30]. Dual effect of PKCδ in β cells apoptosis may attribute to its redistribution between cytosol and nuclear-associated compartment. Nuclear accumulation and activation of PKCδ is required in its pro-apoptotic effect [21], [31], [32]. PKCδ favors apoptotic cell death through inactivation of DNA-dependent protein kinase in the nucleus, which plays a primary role in DNA repair mechanisms [33]. Other nuclear proteins such as protein lamin B, the checkpoint protein hRad9 have been shown to be phosphorylated by PKCδ in genotoxin-treated cells [34], [35]. Recent studies suggested that PKCδ activated the proapoptotic through nuclear accumulation and stimulation of forkhead box class O1 (FOXO1) [22].

RETRACTED

The present study showed that PKCδ was activated and nuclear accumulated in INS-1-TRB3 cells accompanied by TRB3 overexpression. We suggest that PKCδ acts as downstream of TRB3 involved in lipoapoptosis. This hypothesis was further supported by the use of the PKCδ inhibitor rottlerin. Although rottlerin itself has proapoptotic activity as mitochondrial uncoupler [25], attenuation of PKCδ activation prevented INS-1-TRB3 cell apoptosis attributed to TRB3 upregulation, whereas the levels of TRB3 did not change significantly. Since Katrin Eitel et al. concluded that inhibition of PLC blocks FFA-induced PKCδ nuclear translocation [21], we verified the effect of PLC inhibitor in INS-1-TRB3 cells. Likewise, U-73122, a general inhibitor of PLC, lessened the apoptosis restricted to TRB3 overexpression. Although not discussed in detail, TRB3 increases PLC activity, and the following rise in diacylglycerol levels might lead to activation and translocation of PKCδ. Further studies are warranted to delineate the molecular pathway and identify the proteins link the TRB3 with PKCδ, and the study is underway in our lab.

In summary, these studies provide novel insights into the central role of TRB3 in lipoapoptosis in pancreatic β cells. We demonstrated that increased TRB3 expression may explain FFAs-induced β cell apoptosis and implicated the PKCδ pathway in this process for the first time. Inhibition of the TRB3/PKCδ axis could be relevant for preservation of β cell mass and function in conditions associated with increased serum FFA levels. These findings can be incorporated into a new potential therapeutic approach for the treatment of T2DM.

## Materials and Methods

### Ethics statement

The study has been approved by the Committee on the Ethics of Animal Experiments of China-Japan Friendship Hospital (Permit Number: 012#201210). All animal care procedures were in accordance with the Principles of Laboratory Animal Care and the Guide for the Care and Use of Laboratory Animals of the National Institutes. All efforts were made to minimize animal suffering and to reduce the number of the animals used.

### Preparation of palmitate/BSA complex solution

As described previously, palmitate/bovine serum albumin (BSA) conjugates were made by soaping palmitate with NaOH and mixing with BSA [36]. Firstly, a 20 mM palmitate stock solution was prepared in 0.01 M NaOH along with heating at 70°C in a shaking water bath for 30 min. A 5% fatty acid-free BSA solution was prepared in phosphate-buffered saline (PBS) at a 55°C water bath. The palmitate stock solution was mixed with the BSA solution at a 1∶3 volume ratio, and the resulting complex solution contained 5 mM palmitate and 3.75% BSA. The complex solution was diluted in RPMI 1640 (11.1 mM glucose) supplemented with 10% FCS for *in vitro* experiments. The concentration of BSA in 0.2 mM palmitate is 0.15%. For *in vivo* experiments, palmitate/BSA complex solution was not diluted. The mice were injected intraperitoneally with 100 mg/kg palmitate per day.

RETRACTED

### FFA measurement

Mice serum was separated and stored at −20°C immediately until use. The FFA concentrations were assayed following a modified version of the manufacturer's protocol by the nonesterified fatty acid assay kit (Wako Chemicals, Richmond, VA, USA) to accommodate a 96-well microplate.

### Assessment of caspase 3/7 activity

C57BL/6 mice (10–12 weeks old, ∼20 g) were injected intraperitoneally with or without palmitate for 7 days. Then pancreatic islets were isolated as previously described [37]. Apoptosis of islets was determined by Caspase 3/7 activity assays as previously described [38], using Caspase-Glo 3/7 assay according to the manufacturer's instructions (Promega Madison, WI, USA).

### Cell culture

Rat insulin-secreting INS-1 cells (passage 50–90; a gift from Dr Haiyan Wang, University of Geneva, Geneva, Switzerland) [39], [40] and our previously established INS-1-derived stable cell line, TRB3 cells (allowing inducible expression of TRB3) [41] were cultured in RPMI 1640 medium supplemented with 10% (v/v) fetal calf serum (Sigma-Aldrich Company, St. Louis, MO, USA), 50 µM β-mercaptoethanol, 11 mM glucose, 10 mM HEPES, 2 mM glutamine, 1 mM sodium pyruvate, 100 units/ml penicillin, 100 µg/ml streptomycin and incubated at 37°C, 5% CO_2_ as described [40], [41].

### Establishment of INS-1 derived cells permitting inducible expression of TRB3

The stable clone INS-r9 cell line, carrying the reverse tetracycline/Dox-dependent transactivator, was used for the first stable transfection [42]. The plasmid for the second stable transfection was constructed by subcloning cDNA encoding rat TRB3. The inducible TRB3 cells were induced with 500 ng/ml Dox for 48 h as described previously [41], [43]. The TRB3 expression was analyzed by western blot and immunofluorescence.

### RNA interference

The siRNAs of TRB3 was used: 5′-ATC TCT GGC TGC TTC TGC CGA TGT T-3′ and negative control siRNA was used: 5′-UUC UCC GAA CGU GUC ACG UTT-3 (GenePharma, Shanghai, China). The siRNAs were introduced into INS-1 cells by Lipofectamine 2000 (Invitrogen, Paesley, UK). After transfection, cells were cultured for 48 h before treated as indicated.

RETRACTED

### Cell treatment and apoptosis assay

For the TUNEL assay, TRB3 cells were seeded in 96-well plates (5×10^4^ cells per well) and treated with or without 500 ng/ml Dox for 48 h. The cells were then treated with 0.2 mM palmitate/BSA complex or BSA (control) in RPMI 1640 containing 10% FCS for 24 h. In some experiments, the cells were pretreated with or without rottlerin (5 µM Calbiochem, Nottingham, UK) for 1 h or Gö6850 (1 µM Calbiochem, Nottingham, UK) for 1 h before being treated with palmitate. The cells were then washed twice, fixed in 4% paraformaldehyde for one hour, and then permeabilized with 0.1% Triton X-100 in PBS/BSA solution. The TUNEL assay was performed using in situ cell death detection kits (Roche, Indianapolis, IN, USA), according to the manufacturer's protocols.

Caspase-3 activity was measured by caspase-3 assay kit (Molecular Probes, Invitrogen, Carlsbad, CA, USA) following the manufacturer's instruction on harvested cells treated as indicated. Microplate fluorescence reader (Molecular Devices Corp, Sunnyvale, CA, USA) was used for detection.

### Subcellular fractionation and western blot analysis

Radio-immunoprecipitation assay (RIPA) buffer containing protease inhibitors (complete, Mini, Roche Diagnostics Corp., Indianapolis, IN) and phosphatase inhibitors (Phosphatase Inhibitor Cocktail, Cell Signaling Technology, Beverly, MA,USA) was used to isolate total cellular fractions. To evaluate the nuclear PKCδ content, protein lysates were isolated as previously described in detail [44], [45].

Protein levels of lysates were normalized for protein amounts determined by the BCA protein assay kit. Aliquots of 30 µg protein were separated by SDS-polyacrylamide electrophoresis. To verify equal loading and for normalization for quantitation among lanes, immunoblots of the same protein samples were probed for β-actin. The primary antibodies were used at the following dilutions: TRB3 (1∶2500, Calbiochem, La Jolla, CA, USA),PKCδ (1∶1000, Cell Signaling Technology, Beverly, MA), phosphor-PKCδ (1∶1000 Cell Signaling Technologies, New England Biolabs, Hitchin, UK) AKT (1∶1000), p-AKT (1∶1000), and β-actin (1∶5000).

### Subrenal capsular transplantation animal model

Firstly, the 8 week-old nu/nu mice were irreversibly induced to be diabetic by intraperitoneal injection with a relatively high single dose (180 mg/kg) of STZ (Sigma-Aldrich Company, St. Louis, MO, USA). At day 6, TRB3 cells (5×10^6^) were transplanted into the left kidney of STZ-treated diabetic mice to establish the subrenal capsular animal model. The fasting blood glucose began to decline significantly 18 days post-transplantation, and from then on, we injected STZ intraperitoneally once daily with or without palmitate (100 mg/kg per day) and Dox (5 mg/kg per day) for 8 days. All mice were sacrificed at day 32. The left kidneys were immediately fixed in 10% buffer formalin at room temperature overnight and subsequently embedded in paraffin. Sections were then subjected to hematoxylin and eosin (H&E) staining, immunohistochemistry and TUNEL staining.

RETRACTED

### Statistical analysis

The data were expressed as the ± S.E.M. Unpaired two-tailed t-tests were used when the differences between two groups were analyzed. For multiple comparisons between groups, ANOVA followed by Tukey's post-hoc test was used. A *p*<0.05 was considered statistically significant.

## Supporting Information

Figure S1 **INS-1 cell apoptosis was not increased after a 48 h exposure to 500 ng/ml Dox.** INS-1 cells were treated with or without 500 ng/ml Dox for 48 h, and then the cell apoptosis was assessed by TUNEL staining. The bar graph shows the average apoptosis rate, values represent mean ± S.E.M. of three independent experiments, each carried out in triplicate, Scale bar, 50 µm.
(TIF)

Figure S2 **AKT protein phosphorylation in INS-1 derived cells under the indicated treatment.** A representative blot of 3 independent experiments is shown. β-actin was used as a control for protein loading.
(TIF)

Figure S3 **C57BL/6 mice (10–12 weeks old) were intraperitoneally injected with 0.5 ml of 5 mM palmitate, oleate, or BSA (3.75%) per day for 7 days.** We investigated the nuclear translocation (nuclear PKCδ vs. nuclear H1) and activation (phosphorylated PKCδ vs. whole-cell PKCδ) of PKCδ in isolated islets. A representative blot of 3 independent experiments is shown.
(TIF)
